The article "EEG Analysis with Wavelet Transform under Music Perception Stimulation" was retracted in 2023. Reasons: signs of a paper mill; suspected computer-generated content; unreliable results or conclusions; lack of ethics approval or compliance.

# EEG Analysis with Wavelet Transform under Music Perception Stimulation

**DOI:** 10.1155/2021/9725762

**Published:** 2021-12-15

**Authors:** Jing Xue

**Affiliations:** Xi'an University of Posts & Telecommunications, Shaanxi 710000, China

## Abstract

In order to improve the classification accuracy and reliability of emotional state assessment and provide support and help for music therapy, this paper proposes an EEG analysis method based on wavelet transform under the stimulation of music perception. Using the data from the multichannel standard emotion database (DEAP), *α*, *ß*, and *θ* rhythms are extracted in frontal (F3 and F4), temporal (T7 and T8), and central (C3 and C4) channels with wavelet transform. EMD is performed on the extracted EEG rhythm to obtain intrinsic mode function (IMF) components, and then, the average energy and amplitude difference eigenvalues of IMF components of EEG rhythm waves are further extracted, that is, each rhythm wave contains three average energy characteristics and two amplitude difference eigenvalues so as to fully extract EEG feature information. Finally, emotional state evaluation is realized based on a support vector machine classifier. The results show that the correct rate between no emotion, positive emotion, and negative emotion can reach more than 90%. Among the pairwise classification problems among the four emotions selected, the classification accuracy obtained by this EEG feature extraction method is higher than that obtained by general feature extraction methods, which can reach about 70%. Changes in EEG *α* wave power were closely correlated with the polarity and intensity of emotion; *α* wave power varied significantly between “happiness and fear,” “pleasure and fear,” and “fear and sadness.” It has a good application prospect in both psychological and physiological research of emotional perception and practical application.

## 1. Introduction

Music therapy is an emerging discipline integrating music, medicine, psychology, and other fields. It has made some research achievements in the psychological rehabilitation treatment of prenatal education, children's autism, Alzheimer's disease, and other diseases As an important part of social cognition, emotional perception is very important in the process of biological evolution and social interaction in real life [1]. Most neuroscience studies on human emotions use static visual images as stimuli to induce emotions, but in real life, people's emotions can obviously be triggered by many different stimuli. Neuroscience has found that music is also an effective tool for studying emotions [2]. Music has the following advantages: Music can trigger emotional reactions with considerable intensity. These emotions can usually be induced consistently among different subjects. Music not only can arouse unpleasant emotions but also can arouse happy emotions. However, it is difficult to arouse happy emotions through static images [3]. With the development of science and technology and the application of computers, many comprehensive signals are processed by digital signals, which make people's daily working methods reformed. Digital signal processing is generally divided into two categories: steady-state using Fourier analysis and unsteady state (sudden change) using wavelet analysis [4, 5]. Changes in EEG (electroencephalogram) power spectrum are closely related to the polarity and intensity of musical mood; *α* wave power is inversely correlated with brain activity, that is, greater *α* power represents less brain activity, smaller *α* power represents more brain activity, and *α* band power can more to changes in brain behavior than other bands. However, as a new field, the overall EEG research on musical emotion perception is still in the groping stage, looking forward to more and more systematic and detailed research. EEG examination has a significant role in the diagnosis of neurological disease, disease monitoring, and efficacy observation. Abnormal bioelectricity can be found through brain waves, and brain lesions can be detected.

EEG signals can comprehensively reflect the physiological and psychological state of the human body, and it is an effective evaluation method to analyze the emotional state in combination with the changes of EEG signals and then evaluate the effect of music therapy [6]. The activity degree of a certain rhythm wave caused by different emotions is different, so the original signal is decomposed and reconstructed by wavelet transform to obtain the basic rhythm wave. Extracting EEG features of rhythmic waves will be able to better analyze the changes of music emotional EEG [7]. Khaleghi et al. have proposed several linear and nonlinear biomarkers from EEG signals to diagnose ADHD. However, it is still controversial to determine which type of analysis provides us with the best characteristics and biomarkers for diagnosing ADHD. In this study, several kinds of features extracted from EEG for diagnosing ADHD are evaluated and compared. In this study, five types of features are extracted from EEG, including morphology, time, frequency, time-frequency, and nonlinear features. The receiver operates the feature (ROC) curve and the evidence *k* nearest neighbor (EKNN) classifier to determine the efficacy of each feature class in ADHD diagnosis. Statistical analysis showed that 13.15, 13.68, 14.47, 14.03, and 34.73% of the extracted features were significant in morphology, time, frequency, time frequency, and nonlinear domain (*P* < 0.05). The maximum AUC values of five categories such as morphological, temporal, frequency, time frequency, and nonlinear feature are 0.870, 0.796, 0.824, 0.806, and 0.899 [8]. Wavelet packet decomposition reconstruction of affective EEG signals and the *ß* rhythm was used for affective state recognition. The degree of some rhythm wave activity caused by different emotions is different. Therefore, by using the wavelet transform to obtain the basic rhythm wave, the extraction of the EEG features of the rhythm waves will better analyze the changes in the musical mood EEG.

Based on this study, this paper presents an EEG analysis method based on wavelet transformation under music sensing stimulation. The EEG states under different musical stimuli were used as the analysis objects. The frequency band (*α*, *ß*, and *θ*) waves were reconstructed by using the wavelet transform decomposition. Adaptive features based on the EMD make full use of the extracted time-domain waveform features of the rhythmic wave signal (local maximum, minimal, over zero, and mean line). The *α* wave, *ß* wave, and *θ* wave rhythms are decomposed into series of IMF components. Features such as the mean energy and amplitude difference of the IMF were further extracted. Match detection of EEG with various wavelet groups takes the wavelet coefficient and has the minimum variance value. Based on the support vector machine (SVM) classifier for affective state assessment, it then provides help and support for music therapy.

## 2. Research Methods

### 2.1. Algorithm Flow Chart

The general flow of this algorithm is shown in Figure 1.

### 2.2. EMD  Algorithm

EMD is an algorithm for decomposing nonlinear and nonstationary sequence signals based on its own time scale, which is self-adaptive and does not need to set a basis function. The purpose of EMD is to obtain a limited series of IMF components, and the frequency of each IMF component is gradually reduced with the increase of scale, which is helpful to highlight the local part of each component of EEG Features. The EMD principle is as follows, assuming that the original signal is *x* (*t*):

Step 1: find out all local maxima and minima of *x*(*t*) signal.
Step 2: perform curve fitting on all local maximum points in step 1 to form an upper envelope *m*_1_(*t*); all minimum points are fitted into the lower envelope *m*_2_(*t*).
Step 3: find the mean curve *u*(*t*) of the upper and lower envelopes, as shown in the following formula:
  (1) $$\begin{array}{c} u\left(t\right)=\frac{1}{2}\left[m_{1}\left(t\right)+m_{2}\left(t\right)\right]. \end{array}$$
Step 4: separate the envelope mean curve *u*(*t*) from the original signal *x*(*t*) to obtain a residual function *h*_1_(*t*), as shown in the formula:
  (2) $$\begin{array}{c} h_{1}\left(t\right)=x\left(t\right)-u\left(t\right). \end{array}$$
If the residual function *h*_1_(*t*) are satisfied with the following two conditions of the IMF component, such as (1) the difference between the number of zero crossings and the number of extreme points in the whole signal segment is 1 at most, that is, there can be neither a minimum value greater than zero nor a maximum point less than zero in IMF and (2) the upper and lower envelopes of the signal are locally symmetric about the time axis [9]. The residual function *h*_1_(*t*) is the first IMF component; otherwise, *h*_1_(*t*) repeats steps 1–4 as a new original signal and cycle *k* times until the obtained residual function meets the two conditions of the IMF component. At this time, as the first IMF component, the residual function is written as follows:
  (3) $$\begin{array}{c} s_{1}\left(t\right)=h_{1k}\left(t\right). \end{array}$$
This cycle cannot be infinite, and Huang finally gives a component stopping condition similar to the Cauchy convergence criterion, as shown in the following formula:
  (4) $$\begin{array}{c} \text{SD}=\frac{\sum_{t=0}^{T}{\left|h_{k-1}\left(t\right)-h_{k}\left(t\right)\right|}^{2}}{\sum_{t=0}^{T}h_{k-1}^{2}\left(t\right)}. \end{array}$$
When SD is generally 0.1–0.3, the iteration stops, and the screening process ends.
Step 5: put the IMF component *s*_1_(*t*) separated from the original signal *x*(*t*); a residual signal *c*_1_(*t*) is obtained, as shown in the following formula:
  (5) $$\begin{array}{c} c_{1}\left(t\right)=x\left(t\right)-s_{1}\left(t\right). \end{array}$$
Step 6: the residual signal is added. *c*_1_(*t*) repeats steps 1–5 as a new original signal and cycle *n* times until the final residual function is obtained. When *c*_*n*_(*t*) runs as a monotone function or constant, the EMD decomposition process ends, which can be easily obtained from the above formula, as shown in the following formula:
  (6) $$\begin{array}{c} x\left(t\right)=\sum_{i=1}^{n}s_{i}\left(t\right)+c_{n}\left(t\right). \end{array}$$

According to EMD decomposition, the frequency of IMF components in each order is different, and the later the IMF components are separated, the lower the frequency is. Therefore, according to the influence of music on the frequency of EEG rhythm waves, the corresponding features can be extracted from each IMF component.

### 2.3. Feature Extraction

Studies have shown that the EEG characteristics of music-induced emotions are mainly reflected in three rhythm waves: *α*, *ß*, and *θ*. When people are excited, the amplitude of *ß* rhythm increases, while when people are sad, *α* rhythm decreases and *θ* rhythm increases, that is, *θ* rhythm is directly proportional to inhibitory emotion, while *ß* rhythm is directly proportional to stimulating emotion, which is more obvious in the frontal and temporal lobes. Therefore, in this study, F3 and F4 in the frontal region, T7 and T8 in the temporal region, and C3 and C4 in the central region were selected. DEAP database uses a “potency-arousal” two-dimensional emotion model. The emotion model divides emotions into positive and negative poles according to valence. Positive emotions at the positive pole usually bring pleasant feelings, while negative emotions at the negative pole usually produce unpleasant feelings. At the same time, according to arousal, we can distinguish the intensity of emotions. The greater the arousal, the stronger the emotion [9, 10]. Negative emotions generally include sadness, fear, anger, anxiety, pain, and hatred, while positive emotions include happiness, satisfaction, interest, pride, gratitude, and love. In this paper, four common basic emotions are selected, including positive emotions such as happy and exciting and negative emotions such as sad and terrible. No emotion chooses quiet baseline EEG signals [11]. Because 7,680 data points in 60 s are relatively large and MATLAB runs slowly, 1,024 data points are intercepted for analysis. Firstly, 5 kinds of emotional EEG signals of 32 subjects were decomposed and reconstructed into *θ* wave, *α* wave, and *ß* wave by wavelet transform. Taking F4 data in a happy state as an example, its channel reconstruction wave is shown in Figure 2.

The reconstructed three rhythmic waves are decomposed by EMD to obtain IMF components, and the F4 channel data in a happy emotional state can obtain seven IMF components by EMD. Then, the Fourier transform is used to transform into frequency domain, and the frequency spectrum of IMF of each order is obtained.

The frequencies of IMF components obtained by EMD are different, and the higher the order of IMF, the lower its frequency. If all IMF component-related features are extracted, the dimension of the feature vector will be very high. These feature quantities will contain a lot of feature values that have little correlation with music EEG features, which will lead to a decrease in the accuracy of emotion recognition. The frequency of the EEG rhythm wave studied in this paper is 4–30 Hz, so the first three IMF components are intercepted as shown in Figure 3, and these IMF components contain almost 90% of the energy of the signal. The first three IMF components are taken for feature extraction.

As the amplitude of the three rhythmic waves of EEG will change when music intervenes, the amplitude difference of adjacent IMF components is extracted as an eigenvalue, as shown in the following formula:

(7) $$\begin{array}{c} H_{ij}=\frac{1}{n}\left(\sum_{t=1}^{n}\left|s_{i}\left(t\right)-s_{j}\left(t\right)\right|\right), \end{array}$$

where *s*_*i*_(*t*) is the *i*-th IMF component, *s*_*j*_(*t*) is the *j*-th IMF component, *n* is the number of IMF component data points, and *H*_*ij*_ Is the amplitude difference between the *i*-th IMF and the *j*-th IMF component. The frequency difference of each IMF component is large, that is, there is an energy difference, so the average energy of each IMF component is taken as an eigenvalue, as shown in the following formula:

(8) $$\begin{array}{c} {Ε}_{l}=\frac{1}{n}{\sum_{t=1}^{n}\left|s_{l}\left(t\right)\right|}^{2}, \end{array}$$

where *s*_*l*_ is the *l*-th IMF component and *n* is the IMF component data points. El is the average energy characteristic of the *l*-th IMF component. To sum up, a subject in each channel of each type of music in this paper has three kinds of rhythm waves, and each rhythm wave contains three average energy eigenvalues and two amplitude difference eigenvalues, so each subject has 15 eigenvalues.

### 2.4. Lib SVM Classifier

The goal of the SVM classifier is to produce a model based on training data that can be used to predict the target value of test data given only attributes. In this paper, the SVM classification model is selected as C-support vector classification (C-SVC). The basic principle of the C-SVC classification model algorithm: set a given training set as follows: *T*={(*X*_*i*_, *y*_*i*_)*|X*_*i*_ ∈ *R*^*n*^, *y*_*i*_ ∈ {−1,1},  *i*=1,…, *k*}, look for the function *h*(*k*), and use the decision function *y*=*f*(*X*)=sgn(*h*(*x*)) to deduce the output *y* value corresponding to the input vector *x*. The specific steps are as follows:

Step 1: select the appropriate kernel function *K*(*X*_*i*_, *X*_*j*_) and the penalty parameter *c*. The optimization problem is constructed and solved as shown in the following formulas:
  (9) $$\begin{array}{c} \underset{\alpha }{\min}\frac{1}{2}\sum_{i=1}^{k}\sum_{j=1}^{k}y_{i}y_{j}\alpha_{i}\alpha_{j}K\left(X_{i},X_{j}\right)-\sum_{j=1}^{k}\alpha_{j}, \end{array}$$
  (10) $$\begin{array}{c} \text{s.t. }\sum_{i=1}^{k}y_{i}\alpha_{i}=0,0\leq \alpha_{i}\leq C,\;i=1,\ldots ,k. \end{array}$$
Get the optimal solution: *α*^*∗*^=(*α*_1_^*∗*^,…,*α*_*k*_^*∗*^)^*T*^.
Step 2: choose *α*^*∗*^ a component of 0 < *α*_*j*_^*∗*^ < *C* and calculate from it: *b*^*∗*^=*y*_*j*_ − ∑_*i*=0_^*k*^*y*_*i*_*α*_*i*_^*∗*^*K*(*X*_*i*_, *X*_*j*_).
Step 3: construct a decision function, as shown in the following formula:
  (11) $$\begin{array}{c} f\left(X\right)=\mathrm{sgn}\left(\sum_{i=1}^{k}y_{i}\alpha_{i}^{*}K\left(X_{i},X\right)+b^{*}\right). \end{array}$$

In this paper, the Gaussian radial basis function (RBF) is chosen as the kernel function, and its expression is: *K*(*X*_*i*_, *X*_*j*_)=exp(−‖*X*_*i*_ − *X*_*j*_‖/2*σ*^2^), where *σ* is the width parameter.

### 2.5. Wavelet Transform

#### 2.5.1. Selection of Wavelet Bases

The wavelet base treatment analysis and the EEG wavelet coefficient and variance values were calculated. The wavelet bases for multiresolution analysis in continuous wavelet transform include coif system wavelet, rbio wavelet, haar wavelet, db wavelet, wavelet, dmey wavelet, sym wavelet, bior wavelet, and so on, which are the group of wavelet bases that obtained the largest wavelet coefficient and small variance. When the wavelet signal was extracted using wavelet transform, the selection of wavelet base was optimized first.

#### 2.5.2. Multiresolution Analysis

If the six-layer decomposition is performed, the sub-band components of each component correspond roughly one-to-one to low *δ* and high *δ*, *θ*, *α*, *β*, and *γ* in the EEG brain waves. After adopting the six-layer decomposition, the one-to-one corresponding frequency band has a clear physical meaning. Therefore, the original signal *f* (*t*) of EEG was decomposed by six layers, and using the wavelet transform, the wavelet base selection was optimized first. The paper uses the adaptive wavelet base method, matching detection, EEG, and various wavelet bases and takes the wavelet coefficient with the minimum variance value. Therefore, there may be multiple different wavelet bases for the EEG to be analyzed. After multiresolution analysis, obtained coefficients were calculated and classified by SVM.

## 3. Results

### 3.1. No Emotion, Positive Emotion, and Negative Emotion

#### 3.1.1. Distinguish between No Emotion and Positive Emotion

Neuroscientific research on human emotions mostly uses static visual images as stimuli to induce emotions, and real-life human emotions can obviously be triggered by many different stimulus sources. As shown in Table 1, when no emotional state and positive emotions are identified, the average energy and amplitude difference of *ß* waves are higher than the single *α* waves. Moreover, although the optimal accuracy is 100%, the accuracy of the test set is reduced compared with the single *ß* rhythm, indicating that the characteristics of *ß* rhythm waves in EEG signals are related to the positive emotions induced by music and is much better than the classification of mixed waves.

#### 3.1.2. Distinguish between No Emotion and Negative Emotion

As shown in Table 2, it can be seen that when distinguishing between no emotion and negative emotion, alone *α* wave performs better than using *θ* wave alone. The results show that the accuracy of the two kinds of wave mixing features is higher than that of using only one wave, which indicates that the negative emotions induced by music are related to both *α* waves and *θ* waves, but the correlation between *θ* waves and negative emotions is higher than that of *α* waves.

#### 3.1.3. Distinguish between Positive Emotions and Negative Emotions

As shown in Table 3, it can be seen that the accuracy of feature classification between positive emotions and negative emotions is not high, which is similar to that obtained by extracting approximate entropy and wavelet entropy features, mostly in the range of 60–70%. However, the classification accuracy of the features between positive and negative emotions is higher, mostly in 70–80%. Therefore, it is better to use the extracted features of the IMF component of the EEG rhythm wave for classification.

In 1985, Cole and Ray studied the relationship between the high- and low-frequency bands of *ß* rhythm and emotion processing, respectively. The results showed that positive emotion and negative emotion caused different brain activities in the high- and low-frequency bands of *ß* rhythm [12–14]. This study focuses on only one EEG rhythm. After that, Kabuto and Yuan Quan began to study the relationship between the frequency domain characteristics of EEG basic rhythm and music. By analyzing the EEG signal in the happy and relaxed mood induced by music, it was found that the energy of *θ* rhythm wave increased, while the energy of *α* wave decreased obviously [15]. These studies only analyze the relationship between emotion and EEG from a certain rhythm of EEG or only select EEG signals in a certain emotional state as the research object, which lacks universality. In this paper, we choose three kinds of EEG rhythm waves that have a great correlation with emotion and analyze the changes of rhythm waves in the two states of positive emotion and negative emotion and get better classification results, which further expands the research between emotion and EEG [16, 17].

The application field of automatic identification of EEG is not only in the clinical medical diagnosis of epilepsy, encephalitis, Parkinson's disease, Alzheimer's disease, Wilson, brain tumor, epilepsy, arrhythmia, and other diseases but also in the adjuvant treatment of mental trauma, will depression, and so on. When the characteristic waveform is detected, the corresponding intervention treatment can be carried out, and the detection and treatment are automatically intelligent. This paper combines wavelet analysis and empirical mode decomposition to realize the feature extraction of music intervention EEG. The *α*, *β*, and *θ* wave rhythms of EEG were extracted, and according to the characteristics of EEG stimulated by music, 15 characteristic quantities such as amplitude difference of adjacent IMF components and average energy of the first three IMF components were extracted [18]. Pairwise classification of four emotions was solved to some extent. The classification accuracy obtained by this EEG feature extraction method is higher than that obtained by general feature extraction methods and can reach about 70%. However, although the recognition rate of pairwise classification of four emotions has been improved, it cannot achieve the effect of complete separation. For example, the classification effect of sad emotion and terrible emotion is still very low. Therefore, the recognition effectiveness of this feature extraction method between similar emotions needs to be improved [19, 20].

## 4. Conclusion

As an effective emotional inducement source, music has a good application prospect in both psychological and physiological research of emotional perception and practical application. The application field of automatic identification of EEG is not only in the clinical medical diagnosis of epilepsy, encephalitis, Parkinson's disease, Alzheimer's disease, Wilson, brain tumor, epilepsy, arrhythmia, and other diseases but also in the adjuvant treatment of mental trauma, will depression, and so on. When the characteristic waveform is detected, the corresponding intervention treatment can be carried out, and the detection and treatment are automatically intelligent. Especially in recent years, the clinical development of music therapy and brain computer interface in brain neuroscience is very fast, which makes the study of the relationship between music, emotion, and EEG appear more valuable. If the music is arranged according to the law of the emotional response to different music in the EEG rhythm and used for clinical music therapy, its application value is self-evident.

## Figures and Tables

**Figure 1:** Algorithm flow chart.

**Figure 2:** Three rhythmic waves of reconstructed EEG.

**Figure 3:** IMF component spectrogram with determined order.

**Table 1:** Classification of no emotion and positive emotion.

Band	Optimal accuracy rate (%)	Accuracy of test set (%)
*α* wave (N-H)	93.75	84.38
*α* wave (N-E)	96.88	81.25
*β* wave (N-H)	93.75	90.63
*β* wave (N-E)	100.00	100.00
*α* wave + *ß* wave (N-H)	100.00	87.50
*α* wave + *ß* wave (N-E)	100.00	84.38

**Table 2:** Classification of no emotion and negative emotion.

Band	Optimal accuracy rate (%)	Accuracy of test set (%)
*α* wave (N-S)	96.75	93.75
*α* wave (N-t)	93.88	87.50
*θ* wave (N-S)	100.00	93.75
*θ* wave (N-t)	100.00	100.00
*α* wave + *θ* wave (N-S)	100.00	96.88
*α* wave + *θ* wave (N-t)	100.00	100.00

**Table 3:** Pairwise classification between four emotions.

Classify	Approximate entropy + wavelet entropy accuracy (%)	Average energy + amplitude difference (this algorithm) accuracy (%)
H-E	65.63	68.75
H-S	68.75	81.25
E-S	50.00	75.00
H-T	59.38	71.88
E-T	59.38	78.13
S-T	53.13	65.63

## Data Availability

The data used to support the findings of this study are available from the corresponding author upon request.
